# An Efficient Data Classification Decision Based on Multimodel Deep Learning

**DOI:** 10.1155/2022/7636705

**Published:** 2022-05-04

**Authors:** Wenjin Hu, Feng Liu, Jiebo Peng

**Affiliations:** ^1^School of Computer Science, Xi'an Polytechnic University, Xi'an, Shaanxi, China; ^2^Shaanxi Key Laboratory of Clothing Intelligence and Computation, Xi'an, Shaanxi, China

## Abstract

A single model is often used to classify text data, but the generalization effect of a single model on text data sets is poor. To improve the model classification accuracy, a method is proposed that is based on a deep neural network (DNN), recurrent neural network (RNN), and convolutional neural network (CNN) and integrates multiple models trained by a deep learning network architecture to obtain a strong text classifier. Additionally, to increase the flexibility and accuracy of the model, various optimizer algorithms are used to train data sets. Moreover, to reduce the interference in the classification results caused by stop words in the text data, data preprocessing and text feature vector representation are used before training the model to improve its classification accuracy. The final experimental results show that the proposed model fusion method can achieve not only improved classification accuracy but also good classification effects on a variety of data sets.

## 1. Introduction

Text classification originated in the 1950s. From the initial expert-based system to traditional machine learning approaches and now deep learning methods, text classification technology is gradually maturing [1]. In recent years, deep learning has been a hot topic in academic research. Great breakthroughs have been made in various fields by using deep learning technology, such as natural language processing, computer vision, and reinforcement learning. Text classification based on deep learning is both a trending subject and a long-term challenge for researchers.

In a study on text classification, Rocchio [2] first proposed the Rocchio text classification algorithm, which uses a training set to construct a prototype vector for each class and allocates an input document to a certain class by calculating the similarity between all documents in the training set and the prototype vector. This method is easy to implement and calculate. However, it does not perform well in tasks with multiple categories and is mostly suitable for document classification problems with fewer categories. Based on the Rocchio algorithm, Somya and Srinivasa [3] proposed a Rocchio algorithm with a hierarchical structure. This algorithm adopts the term frequency-inverse document frequency (TF-IDF) feature extraction method to conduct large-scale multilabel text classification for hierarchical data sets and has a good classification effect on such data sets. However, it has poor performance on multitype data sets. Schapire [4] first proposed the boosting classification algorithm based on the idea of model fusion. This algorithm mainly fuses multiple weak learners into a strong learner, achieving an improved classification effect; then, he proposed the bagging algorithm [5]. Among these weak learners, random forests, boosting trees, and gradient boosting decision trees (GBDTs) [6] are the basic models used when combining decision trees with boosting and bagging algorithms; this approach provides a significantly improved classification effect. Based on the idea of boosting, Bloehdorn and Hotho [7] proposed an adaptive boosting algorithm with semantics. The model algorithm uses an integrated learning method to improve the stability and accuracy of text classification. However, the number of trained models is large; the calculations are very complicated; and the interpretability between models is reduced. Kowsari [8] and others proposed a random multimodel classification method, which uses the network learning architectures of a deep neural network (DNN), recurrent neural network (RNN), and convolutional neural network (CNN) to randomly generate numbers of hidden layers and neurons for each model and obtain predictions through majority voting. As a result, this method has achieved improved text classification accuracy. However, since the numbers of hidden layers and neurons are randomly generated, the network structure generated each time is different, making the model training process difficult and the calculations very complicated. References [9–11] proposed a widely used Bayes classifier, which is a single classifier. It has a good classification effect on text data, and the calculations are fast and easy to implement. However, the Bayesian classifier performs poorly on text with sparse data. Therefore, Kim et al. [12] developed a method and a strong data distribution assumption to alleviate the problem regarding poor prediction for sparse data and solve the poor classification problem for sparse text data. Another powerful classifier is the support vector machine (SVM) [13], which uses a flexible and diverse kernel method to project data into a high-dimensional space, thereby using the hyperplane in the high-dimensional space to classify the data; the classification effect of this method is relatively good, but the effect of a single classifier is reduced when used on multiple data sets.

The traditional single classifier, which can be used to achieve good classification results, is used to train the network model for a specific data set. While the single classifier cannot handle various data sets, the integrated model can solve the problem of accuracy under various data sets, but the training of the integrated model is complex and time-consuming. The traditional single classification model and integrated model are improved in this paper, and the data sets are trained by combining multiple network models. First, a variety of optimizer algorithms are used to address text feature problems such as long texts and sparse texts. Second, the learning rate in the training process of the model is adjusted by the optimizer so that the trained model can handle data sets with different text characteristics and increase the flexibility of the model.

Improvements are made on the basis of three network architectures: DNN, RNN, and CNN. In the DNN network architecture, the BP algorithm and many optimizer algorithms are combined to train the model. In the RNN network architecture, the GRU [14] network with horizontal and vertical learning, multiple optimizer algorithms, and the ReLU [15] activation function training model are designed. In the CNN network architecture, multilayer convolution and pooling are used to extract text features and combined with a variety of optimizer algorithms [16] to train the model. Finally, the improved network architectures are used to obtain a powerful text classification model by using a fusion strategy and parallel training method.

## 2. Materials and Methods

The text classification process in this paper includes the following steps: text data preprocessing, text vector representation, text feature extraction, optimizer selection, model design, model fusion, and model evaluation.  Figure 1 shows the flowchart of the proposed method from preprocessing to model evaluation. The following describes the detailed process of the whole text classification in this article.

### 2.1. Text Preprocessing

The main purpose of text preprocessing is to clean the original text data. Most text and document data sets contain many unnecessary words, such as stop words, spelling errors, and slang. When determining word frequency statistics, these noisy data and unnecessary features adversely affect the performance of the models and the classification results. In this paper, the stop vocabulary list in the NLTK corpus is incorporated for word removal and processing. Additionally, regular expressions are used to remove spaces and some special characters to reduce the calculation cost and classification error of the model training.

### 2.2. Word Representation

Word representation converts a text string into a numerical vector that can be processed by a computer. The commonly used text vector representation methods are the bag-of-words [17] method, word2vec [18], and the GloVe [19] method. This paper uses the GloVe model for text vector representation. The basic idea is to construct a co-occurrence matrix through a corpus and then learn word vectors based on the co-occurrence matrix and the GloVe model. The model uses matrix decomposition with latent semantic analysis (LSA) derived global features and word2vec local context information to transform the matrix. Together, this approach not only realizes the global statistical features in the corpus but also uses local context features to represent vectors. When using the GloVe model for training, the word vector for the given text is calculated by introducing a loss function such as

(1) $$\begin{array}{c} J=\sum_{i,j}^{N}f\left(X_{i,j}\right){\left(\upsilon_{i}^{T}\upsilon_{j}+b_{i}+b_{j}-\log\left(X_{i,j}\right)\right)}^{2}, \end{array}$$

where *υ*_*i*_ and *υ*_*j*_ are the word vectors of word *i* and word *j*, respectively; *b*_*i*_ and *b*_*j*_ are bias terms; *f* is a weight function; log(*X*_*i*,*j*_) represents the number of times word *j* appears in the context of word *i*; *N* is the size of the vocabulary; and *N∗N* is the dimensionality of the co-occurrence matrix. Additionally, the weight function of *f* is defined; this is done to prevent some weights from being too large. Additionally, some weights are too small, which affects the text classification accuracy, so function *f*(*x*) is defined as follows:

(2) $$\begin{array}{c} f\left(x\right)=\left\{\begin{array}{cc} {\left(\frac{x}{x_{\max}}\right)}^{\alpha }, & x<x_{\max},\\ 1, & \text{Other.} \end{array}\right) \end{array}$$

### 2.3. Feature Extraction

The commonly used feature extraction methods are TF-IDF [20] and *N*-gram [21]. When TF-IDF is used to extract text features, the sequence relationship between words cannot be captured, so the features of the text cannot be fully extracted. Therefore, this paper uses the *N*-gram method to extract text features. In text data, a sequence or a sentence is composed of *m* words. Then, the probability of the occurrence of the *m*-th word is related to the previous *m* − 1 words, and the probability value *p* (*w*_1_, *w*_2_,…, *w*_*m*_) is calculated. According to the chain rule, the final calculation result is shown in the following equation:

(3) $$\begin{array}{c} p\left(w_{1},w_{2},\ldots ,w_{m}\right)=p\left(w_{1}\right)*p\left(w_{2}|w_{1}\right)*\\ p\left(w_{3}|w_{1},w_{2}\right)\ldots p\left(w_{m}|w_{1},\ldots w_{m-1}\right) \end{array}$$

Compared with a 1-gram and a 2-gram, the *N*-gram method provides extracted text features that can detect more information.

### 2.4. Optimizer Algorithm

#### 2.4.1. An Optimization Algorithm for Vibration Reduction Based on RMSProp

When training the parameters of the model, the choice of the learning rate affects the efficiency and performance of the model. If the learning rate is too large, violent oscillations will occur when calculating the gradient, resulting in failure to converge to the global optimal solution, and if the learning rate is too small, the training speed will become very slow. The current method is the simulated annealing algorithm. When training model parameters, a threshold is defined for the learning rate change range, and the learning rate is adjusted. However, this approach requires a threshold to be defined in advance, and it cannot adapt to changing text data types. To solve the problem regarding learning rate threshold changes and oscillations, this paper uses the RMSProp algorithm based on Nesterov momentum. The algorithm first initializes the learning rate and continuously dynamically updates the learning rate during the training process to prevent this rate from being excessive or small during the training process, as this would affect the training results. The specific main steps are as follows. First, a minibatch containing *m* samples from the training set is formed, and the gradient sum and average of these small samples are calculated, as in equation (4). At the same time, an exponential decay coefficient such as equation (5) is used to control the amount of historical information, that is, the cumulative gradient, to dynamically update the size of the learning rate (equation (6)) and the model parameters (equation (7)).

(4) $$\begin{array}{c} g=\frac{1}{m}\nabla_{\tilde{\theta }}\sum_{i}ℒ\left(f\left(x^{\left(i\right)};\tilde{\theta }\right),y^{\left(i\right)}\right), \end{array}$$

(5) $$\begin{array}{c} r=\rho r+\left(1-\rho \right)g*g, \end{array}$$

(6) $$\begin{array}{c} \upsilon =\alpha \upsilon -\frac{\varepsilon }{\sqrt{r}}*g, \end{array}$$

(7) $$\begin{array}{c} \theta =\theta +\upsilon , \end{array}$$

(8) $$\begin{array}{c} \tilde{\theta }=\theta +\alpha \upsilon , \end{array}$$

where *r* represents the exponential decay coefficient, *υ* represents the update of the calculation speed, *θ* represents the update of the parameters, *g* represents the gradient, and *α* represents the momentum coefficient. At the same time, to reduce the violent oscillations observed when training the model parameters, an idea based on Nseterov momentum is adopted, and a momentum coefficient is added before calculating the gradient to slow the oscillations, as shown in equation (8). Therefore, the optimizer of the RMSProp algorithm combined with Nesterov momentum improves the training speed and accuracy of the model.

#### 2.4.2. An Optimal Deviation Correction Algorithm Based on Adam

Adam is a simple and computationally efficient optimization algorithm that can overcome the problems encountered in large data sets and high-dimensional parameter spaces. Among traditional classification methods, such as naive Bayes classifiers and SVMs, for text data with large data sets, it is necessary to consider the memory consumption of the naive Bayes model training process and the model oscillation problem, while SVMs do not possess this problem. A kernel method puts text data into a high-dimensional space, and the resulting model has many parameters and is highly complicated to calculate. Therefore, the Adam algorithm with deviation correction is introduced to solve the shortcomings of traditional methods. The basic idea is that when Adam calculates the gradient, it introduces the first-order moment estimation (equation (9)) and the second-order moment estimation (equation (10)) and then corrects the deviation of the first-order moment (equation (11)) and that of the second-order moment (equation (12)) to address gradient sparseness and unevenness. Equation (9) updates the first-order moment by calculating the gradient *g* and the exponential decay rate *ρ*_1_ and simultaneously corrects the deviation through equation (11), speeding up the convergence of the model. Equation (10) introduces the second-order moment, and equation (12) corrects the deviation to improve the model's ability to deal with nonstationary targets. At the same time, the Δ*θ* parameter (equation (13) is used to update the value of parameter *θ* in equation (14)). This paper uses the aforementioned algorithm in text classification to train the model parameters to reduce memory consumption and simultaneously solve the problem of convex model convergence.

(9) $$\begin{array}{c} s=\rho_{1}s+\left(1-\rho_{1}\right)g, \end{array}$$

(10) $$\begin{array}{c} r=\rho_{2}r+\left(1-\rho_{2}\right)g*g, \end{array}$$

(11) $$\begin{array}{c} \hat{s}=\frac{s}{1-\rho_{1}^{t}}, \end{array}$$

(12) $$\begin{array}{c} \hat{r}=\frac{r}{1-\rho_{2}^{t\;}}, \end{array}$$

(13) $$\begin{array}{c} \Delta \theta =-\varepsilon \frac{\hat{s}}{\delta +\sqrt{\hat{r}}}, \end{array}$$

(14) $$\begin{array}{c} \theta =\theta +\Delta \theta , \end{array}$$

where *s* represents the first-order moment, *g* represents the value of the sample gradient, *ρ*_1_ and *ρ*_2_ represent the estimated exponential decay rate, *θ* represents the parameter calculated by the model, *δ* represents a small constant used for numerical stability, *ε* represents the step size, and Δ*θ* is used to update the parameter *θ*.

#### 2.4.3. An Improved Optimization Algorithm Based on SGD

Before the introduction of the SGD algorithm, the most commonly used gradient algorithm was the batch gradient descent (BGD) algorithm, which is aimed at an entire data set and calculates the gradient direction for all samples. Although this method can obtain the global optimal solution, when the amount of data is large, the number of required calculations is large, and the calculation speed is slow. To overcome the shortcomings of the BGD method, this paper uses the SGD algorithm. SGD is a widely used optimization algorithm. It is an improvement over the classic gradient descent algorithm. The basic idea is that all training data can be obtained from the training data in each iteration. A random sample is taken to estimate the gradient of the objective function, so the time complexity of the algorithm is greatly reduced, and this approach is applied to large-scale text data sets. When using the SGD algorithm in this paper, a set of text training data is input into the model. The objective function is calculated as follows:

(15) $$\begin{array}{c} \underset{w\in {\mathbb{R}}^{n}}{\min}F\left(w\right)=\frac{1}{m}\sum_{i}ℒ\left(f\left(x^{\left(i\right)};w\right),y^{\left(i\right)}\right), \end{array}$$

where ℒ represents the experience loss of the model *f*(*x*^(*i*)^; w); the model parameter values are calculated as follows:

(16) $$\begin{array}{c} w=\frac{1}{m}\sum_{i}^{m}w_{i}-\eta_{i}\nabla ℒ\left(f\left(x^{\left(i\right)};w_{i}\right),y^{\left(i\right)}\right). \end{array}$$

### 2.5. Model Structure and Fusion

#### 2.5.1. DNN Architecture

The DNN structure in this paper is designed with an input layer, a hidden layer, and an output layer, as shown in Figure 2. The input layer is the processed text feature vector, and the ReLU activation function is used in the hidden layer (as in equation (17)) to reduce the required number of calculations when using the backpropagation algorithm to update the parameters. At the same time, the dropout algorithm is introduced to solve the problem of gradient disappearance in the training process, and finally, the softmax function, such as equation (18), is used to solve the multiclassification problem when outputting.

(17) $$\begin{array}{c} f\left(x\right)=\max\left(0,x\right), \end{array}$$

(18) $$\begin{array}{c} \text{Softmax}\left(z_{i}\right)=\frac{e^{z_{i}}}{\sum_{c=1}^{C}e^{z_{c}}}, \end{array}$$

where *z*_*i*_ represents the output value of the *i*-th node and *c* is the number of output nodes.

#### 2.5.2. RNN Architecture

To solve the information loss problem in the traditional RNN network propagation process, the gate structures of LSTM [22] and GRU networks are generally used to retain important information. Because the network parameters of GRU are less than those of LSTM, the gradient disappearance problem can be prevented and reduce the computational complexity and the overfitting of the training data. The GRU network design unit is shown in Figure 3. This method uses a gating mechanism, which contains an update gate and a reset gate. The calculations are shown in equations (19) and (20), and the output vector is calculated via equations (21) and (22). The final RNN architecture is shown in Figure 4. Each GRU unit in the network can learn not only horizontally but also longitudinally to reduce the information loss problem in the communication process.

(19) $$\begin{array}{c} z_{t}=\sigma \left(W_{z}*\left[h_{t-1},x_{t}\right]\right), \end{array}$$

(20) $$\begin{array}{c} r_{t}=\sigma \left(W_{r}*\left[h_{t-1},x_{t}\right]\right), \end{array}$$

(21) $$\begin{array}{c} {\tilde{h}}_{t}=\tan\text{h}\left(W*\left[h_{t-1}*r_{t},x_{t}\right]\right), \end{array}$$

(22) $$\begin{array}{c} h_{t}=\left(1-z_{t}\right)*h_{t-1}+z_{t}*{\tilde{h}}_{t}, \end{array}$$

where *z*_*t*_ represents the update gate vector at time *t*, *x*_*t*_ represents the input text feature vector, *𝒲* represents the parameter matrix, *σ* represents the ReLU activation function, *r*_*t*_ represents the reset gate vector, and *h*_*t*_ represents the output vector.

#### 2.5.3. CNN Architecture

CNNs were originally used to address image problems, but in natural language processing, the use of CNNs for text classification has achieved better results. In this paper, when the CNN is used for text classification, a six-layer convolution layer and a maximum pooling layer are used, as shown in Figure 5. The model adopts one-dimensional convolution. Without changing the width of the text sequence, the pooling layer uses the maximum pooling strategy to continuously extract important features from the text data through one-dimensional convolution and maximum pooling and then uses a pooling layer to combine the gathered text feature information and input it into the fully connected layer. Finally, the category information of the classified text is output.

#### 2.5.4. Model Fusion

Commonly used model fusion strategies include the averaging method, stacking method, and majority voting method. The main idea of the averaging method is to average the prediction results of each model and use the average value as the final prediction result. The stacking method uses model cross-validation, combining the features between models and training the newly combined features into a new model. Through this repeated feature stacking method, a strong classifier is finally obtained. The method of majority voting involves calculating the statistics of the classification results of each classifier. Among them, the classifier with the most votes divides the final data points in the corresponding category. This method is simple to calculate and easy to implement, and the classification effect is better than that of a single classification approach. The whole model fusion process is shown in Figure 6. The fusion steps of the entire model can be seen in Figure 6; first, the text data set is preprocessed, and the features are extracted and converted into a matrix (*x*_1_, *x*_2_, *x*_*m*−1_, and *x*_*m*_). Then, the text feature vector is input into the designed network architecture for parallel training, and each network architecture uses different optimization algorithms. A total of *n* models are calculated; then these *n* models are tested in parallel on the test sets to obtain the prediction results of each model; and finally, these *k* results are selected through the fusion strategy to select the final prediction result as the classification result of this mode.

Based on the above fusion strategy, the main idea is as follows: the total number of models trained in parallel is *k*, the number of document categories is *m*, and the classification results of each model for text data *i* are counted. Among them, the text data *i* with the most votes is considered to belong to category *c*_*ij*_. Finally, the accuracy rates belonging to category *c*_*ij*_ are summed and averaged as the final prediction result, and the calculations are shown in the following equations:

(23) $$\begin{array}{c} y_{ij}=\left[y_{i1},y_{i2}\ldots ,y_{ik}\right], \end{array}$$

(24) $$\begin{array}{c} c_{ij}=\max\left[c_{i1},c_{i2},c_{i3}\ldots ,c_{im}\right], \end{array}$$

(25) $$\begin{array}{c} {\hat{p}}_{ij}=\frac{\sum_{n=1}^{N}\text{softmax}\left(y_{in}\right)}{N}, \end{array}$$

where *y*_*ij*_  represents the result of model *j* for the classification of text *i*, *k* represents the number of training models, *m* represents the number of categories in the document, *c*_*im*_ represents the number of votes stating that text data *i* belongs to category *m*, ${\hat{p}}_{ij}\;$ represents the number of text data *i* belonging to the accuracy of category *j*, and *N* represents the number of votes.

## 3. Results and Discussion

### 3.1. Datasets

To verify that the fused model has generalizability, this paper uses three different data sets, as shown in Table 1: 20Newsgroups, Reuters, and Web of Science. The 20Newsgroups data set is mainly composed of 20 newsgroups for different topics. It contains 20,000 document data. The Reuters news data set contains 21,578 document data and a total of 90 categories. The Web of Science data set is a collection of academic article abstracts. The data sets include WOS5736 and WOS11967. This paper uses 80% of the documents as training data and 20% as test data. The relationships are shown in Table 1.

### 3.2. Evaluation

This paper uses accuracy, recall, and *F*_1−score_ to measure the classification performance of the model. The calculation equations are as follows:

(26) $$\begin{array}{c} \text{Accuracy}=\frac{\left(\text{TP}+\text{TN}\right)}{\left(\text{TP}+\text{FP}+\text{FN}+\text{TN}\right)}, \end{array}$$

(27) $$\begin{array}{c} \text{Recall}=\frac{\text{TP}}{\text{TP}+\text{FN}}, \end{array}$$

(28) $$\begin{array}{c} F1_{\text{score}}=\frac{2\text{TP}}{2\text{TP}+\text{FP}+\text{FN}}. \end{array}$$

### 3.3. Parameter Settings

This paper uses the GloVe model to learn word vectors, as this model can realize global feature statistics in the corpus and local context feature vectors. At the same time, to prevent the overfitting of the training data, the dropout value is set to 0.5 in each network architecture. Each architecture model uses Adam, SGD, and RMSProp as three optimization algorithms and the ReLU activation function to improve the training speed of the model. The specific parameters are shown in Tables 2–4.

### 3.4. Experimental Results

To verify the classification performance of the proposed multimodel fusion approach and show that it is better than other single classification models, the experimental results obtained on three different public data sets are compared. The results are shown in Table 5.

Table 5 shows the classification results of the majority votes for nine models on the data sets. On the Reuters data set, the voting classification accuracy of the nine models reaches 89.23%, which is 0.66% higher than the model with the highest accuracy in the comparative experiments. The testing results of the fusion model are shown in Figure 7, and the comparative results of the four models are shown in Figure 8. On the 20Newsgroups data set, when training the fusion model, 100 epochs are required for convergence, and the classification accuracy of the models reaches 88.87%, which is 5.13% higher than the model with the highest accuracy in the comparative experiments. The testing results of the fusion model and comparative models are shown in Figures 9 and 10, respectively. The classification accuracy rate that is achieved by the proposed models on the WOS5736 data set is 92.33%, which is 0.35% higher than the model with the highest accuracy in the comparative experiments. The testing results of the fusion model and comparative models are shown in Figures 11 and 12, respectively. The classification accuracy rate of the proposed models on the WOS11967 data set is 85.08%, which is 1.11% higher than the model with the highest accuracy in the comparative experiments. The testing results of the fusion model and comparative models are shown in Figures 13 and 14, respectively. Additionally, on four data sets, the recall and *F*1_score_ of the fusion model are higher than DNN, RNN, and CNN models. In summary, the model fusion method used in this paper has a better classification effect than a single classifier, and the fusion model has a more generalizable effect, which is specifically manifested as not only a better classification effect on a data set but also a good classification effect on a variety of data sets.

## 4. Conclusion

A new classification method is proposed in this paper to solve the problems of data sets and the accuracy of a single model. The combination of parallel training of multiple deep learning architectures and integrated strategies is used to obtain the model. To verify the efficiency of the fusion model, the experimental evaluation of the fusion model on the Reuters, 20Newsgroups, WOS5736, and WOS11967 data sets shows that the accuracy, recall, and *F*1_score_ are higher using the fusion model compared with the DNN, RNN, and CNN models. The results show that the fusion model can also improve text classification and an integration strategy can be used to provide flexibility for classification. This model also provides a new text classification method, which can be applied to a wide range of data sets. In future research, we will further explore the network structure of the fusion model and the influence of each network parameter on the classification results and analyze whether a shallow model can be used to improve the accuracy of the ultimate model while increasing training speed.

## Figures and Tables

**Figure 1:** Overview of the text classification pipeline.

**Figure 2:** DNN architecture.

**Figure 3:** GRU network.

**Figure 4:** RNN architecture.

**Figure 5:** CNN architecture.

**Figure 6:** Model fusion structure.

**Figure 7:** Reuters accuracy function for multimodel deep learning (MDL) trained by nine models in this paper.

**Figure 8:** Reuters accuracy function for a comparative experiment in this paper.

**Figure 9:** 20Newsgroups accuracy function for multimodel deep learning (MDL) trained by nine models in this paper.

**Figure 10:** 20Newsgroups accuracy function for a comparative experiment in this paper.

**Figure 11:** WOS5736 accuracy function for multimodel deep learning (MDL) trained by nine models in this paper.

**Figure 12:** WOS5736 accuracy function for a comparative experiment in this paper.

**Figure 13:** WOS11967 accuracy function for multimodel deep learning (MDL) trained by nine models in this paper.

**Figure 14:** WOS11967 accuracy function for a comparative experiment in this paper.

**Table 1:** Types of datasets.

Datasets	Training (%)	Testing (%)	Categories
20Newsgroups	80	20	20
Reuters	80	20	90
WOS5736	80	20	11
WOS11967	80	20	35

**Table 2:** DNN model parameters.

Parameter	Value
Word vector dimension	100
Learning rate	0.001
Hidden layers	6
Dropout	0.5
Activation function	ReLU
Hidden layer size	512
Batch size	64
Maximum number of words in text	500

**Table 3:** RNN model parameters.

Parameter	Value
Word vector dimension	100
Learning rate	0.001
Hidden layers	4
Dropout	0.5
Activation function	ReLU
Hidden layer size	64
Batch size	64
Maximum number of words in text	500

**Table 4:** CNN model parameters.

Parameter	Value
Word vector dimension	100
Learning rate	0.001
Convolutional layer	6
Flatten layer	1
Pooling layer	6
Fully connected layer	2
Activation function	ReLU
Dropout	0.5
Batch size	64
Maximum number of words in text	500

**Table 5:** Result comparison for text classification (unit %).

	Reuters			20Newsgroups			WOS5736			WOS11967		
	Acc	Recall	F1	Acc	Recall	F1	Acc	Recall	F1	Acc	Recall	F1
DNN	84.82	83.42	82.75	83.74	82.23	81.15	90.59	87.45	86.36	82.37	80.56	79.73
RNN	88.57	86.16	85.78	82.08	80.82	80.34	91.98	89.67	89.05	84.59	83.52	83.87
CNN	84.92	82.63	82.02	80.21	80.13	79.49	91.28	90.31	89.72	82.95	80.65	80.38
This paper	89.23	88.45	88.28	88.87	87.92	86.88	92.33	91.10	90.66	85.08	84.32	84.98

## Data Availability

Three types of data sets from different pages include the following. 20Newsgroups data set contains 20,000 documents with 20 categories. Reuters data set contains 21,578 documents with 90 categories. The Web of Science data set contains WOS11967 and WOS5736. WOS11967 contains 11,967 documents with 35 categories, which include 7 parents categories. WOS5736 contains 5,736 documents with 11 categories, which include 3 parents categories. These links are provided in these statements. All links are given below: (1) https://archive.ics.uci.edu/ml/machine-learning-databases/20newsgroups-mld/, (2) http://kdd.ics.uci.edu/databases/reuters21578/reuters21578.html, and (3) https://data.mendeley.com/datasets/9rw3vkcfy4/2.
